# SHAKF-PU: Sage–Husa Adaptive Kalman Filtering-Based Pedestrian Characteristic Parameter Update Mechanism for Enhancing Step Length Estimation in Pedestrian Dead Reckoning

**DOI:** 10.1155/2024/1150076

**Published:** 2024-02-08

**Authors:** Chinyang Henry Tseng, Jiunn-Yih Wu

**Affiliations:** ^1^Department of Computer Science and Information Engineering, National Taipei University, New Taipei City, Taiwan; ^2^College of Medicine, Chang Gung University, Taoyuan, Taiwan; ^3^Department of Emergency Medicine, Chang Gung Memorial Hospital, Keelung, Taiwan

## Abstract

Step length estimation (SLE) is the core process for pedestrian dead reckoning (PDR) for indoor positioning. Original SLE requires accurate estimations of pedestrian characteristic parameter (PCP) by the linear update, which may cause large distance errors. To enhance SLE, this paper proposes the Sage–Husa adaptive Kalman filtering-based PCP update (SHAKF-PU) mechanism for enhancing SLE in PDR. SHAKF has the characteristic of predicting the trend of historical data; the estimated PCP is closer to the true value than the linear update. Since different kinds of pedestrians can influence the PCP estimation, adaptive PCP estimation is required. Compared with the classical Kalman filter, SHAKF updates its *Q* and *R* parameters in each update period so the estimated PCP can be more accurate than other existing methods. The experimental results show that SHAKF-PU reduces the error by 24.86% compared to the linear update, and thus, the SHAKF-PU enhances the indoor positioning accuracy for PDR.

## 1. Introduction

Pedestrian dead reckoning (PDR) [1] is designed for indoor positioning while pedestrians walking dynamically. PDR collects the pedestrian walking movement data, called pedestrian characteristic parameter (PCP), such as acceleration, gyroscope, and magnetometer. PDR utilizes PCP to perform step length estimation (SLE) to achieve indoor positioning. The original PCP is an empirical value, so cumulative errors occur over update periods.

To avoid cumulative errors, a dead reckoning algorithm based on Bluetooth and multiple sensors (DRBM) [2] establishes the positioning observation intervals for SLE by the initial and final positions based on the timing of the maximum received signal strength indication (RSSI). In each interval, DRBM updates PCP in real time instead of a fixed value to avoid cumulative errors. To update PCP, DRBM adopts a linear update, which directly updates PCP for the next interval. However, the PCP in each interval can be different, and positioning errors occur for DRBM.

The classical Kalman filter (CKF) is a popular approach to estimating suitable PCP in each interval [3–5]. Several works adopt an extended Kalman filter (EKF) to estimate the acceleration [6–8] for SLE in PDR. However, the acceleration can be very dynamic, so the PCP estimation by CKF can be used without focusing on the acceleration and velocity by EKF [3–5].

For pedestrians having different heights, walking speeds, and terrain, their step lengths are different. CKF in DRBM estimates the step length for the current pedestrian in the experiment and utilizes linear updates to estimate the length in each positioning interval. For different pedestrians, CKF can estimate their steps. Although DRBM assumes the pedestrians walk in a constant pattern, the walking styles of different kinds of pedestrians can influence their PCP estimations in each interval. The adaptive PCP estimation in each interval is required, and the linear update in DRBM is insufficient.

Besides, CKF and EKF usually adopt two fixed empirical parameters, *Q* and *R*. To achieve adaptive *Q* and *R* in each positioning interval, the Sage–Husa adaptive Kalman filter (SHAKF) is an ideal solution, and many related applications adopt SHAKF to estimate their core parameters [9–14]. These applications show the SHAKF can adaptively estimate core parameters in real time. Thus, SHAKF is ideal for estimating PCP for SLE but is not adopted in current PDR-related works.

Therefore, this paper proposes a SHAKF-based PCP update (SHAKF-PU) mechanism for SLE in PDR. SHAKF can estimate PCP based on adaptive *Q* and *R* in each positioning interval of PDR instead of static linear update in DRBM. Since SHAKF can adaptively estimate PCP for different kinds of pedestrians, SHAKF performs better PCP updates than CKF. As the experiment results, SHAKF-PU enhances the step estimation accuracy and reduces the indoor position errors based on SHAKF.

The remainder of this paper is organized as follows: Section 2 introduces the related works for PDR, CKF, SHAKF, and their applications.  Section 3 introduces SLE, which is the enhancement target for SHAKF-PU.  Section 4 shows the proposed SHAKF-based PCP update mechanism.  Section 5 illustrates the enhanced SLE based on SHAKF-PU.  Section 6 shows the experiment results of SHAKF compared with the other PCP update methods.  Section 7 concludes the work.

## 2. Related Works

To avoid cumulative errors, dead reckoning is an ideal approach for PDR. DRBM [2] establishes the positioning intervals with or SLE by the initial and final positions based on the timing of the maximum RSSI. While the pedestrian enters the initial position and leaves the final position, a positioning interval occurs with several steps for SLE. In the interval, SLE requires PCP collected during the interval for indoor positioning. Thus, PCP update is critical for SLE, and DRBM adopts linear update, which uses the current PCP for the next interval.

Kalman filter is a popular approach for SLE [3–5]. These three works adopt the CKF as their zero-velocity update for SLE to resist dynamic changes of acceleration. On the other hand, several works [6–8] adopted an EKF to deal with the acceleration for SLE in PDR. For these works, collecting reliable acceleration data values is challenging, though they use EKF to resolve this issue.

For both CKF and EKF, they use static *Q* and *R* values to estimate the errors of each estimation interval. SHAKF provides adaptive *Q* and *R* values, which can be adjusted by historical values in each estimation interval. Thus, SHAKF is adopted in many applications [9–14], such as frequency scanning interferometry [9], motor sensor position [10], slop estimation [11], strapdown inertial navigation [12], radar target tracking [13], and vessel path-following control [14]. These applications require estimating critical values in real time from a noisy environment. SHAKF can reflect the real-time offsets by adaptive *Q* and *R* values, so SHAKF is a better choice than CKF and EKF. However, SHAKF is not adopted in PDR for SLE, especially for PCP updates. Thus, this work adopts SHAKF for better PCP update estimation for enhancing SLR in PDR.

## 3. SLE

In SLE for PDR [2], two Bluetooth chips are set up, one as the reference point for the starting point and the other as the reference point for the endpoint. The user holds the sensor and walks from the start point to the endpoint. The sensor provides ground vertical acceleration values, and the Bluetooth chips provide the respective RSSI values. The ground vertical acceleration calculates the step length through the SLE formula as follows [2]:

(1) $$\begin{array}{c} L=s\times \sqrt[{4}]{a_{\text{max}}-a_{\text{min}}}. \end{array}$$

In Equation (1), *L* is the step length, *s* is the PCP value, *a*_max_ is the maximum ground vertical acceleration, and *a*_min_ is the minimum ground vertical acceleration.

To define a step length segment from the ground vertical acceleration, it is necessary to set up a high threshold and a low threshold for the acceleration. When the ground vertical acceleration is higher than the high threshold, the state value is 1. When the ground vertical acceleration is between the high threshold and the low threshold, the state value is 0. When the ground vertical acceleration is below the low threshold, the state value is −1.

The process of state value going through 1 → 0 → −1 → 0 → 1 is defined as one step, as shown in Figure 1. According to Equation (1), *a*_min_ is the minimum ground vertical acceleration when the step is at the state value −1, and *a*_max_ is the maximum ground vertical acceleration when the state value is at 1.

The original values of the ground vertical acceleration may involve the noise, so the periodicity is not obvious. Therefore, an average filter is needed to reduce the noise. When the ground vertical acceleration is processed by the average filter, its periodicity becomes obvious, which helps split the step length.

PDR needs to have an initial position reference. When the RSSI reaches its maximum value, the pedestrian position is closest to the reference point. In other words, when the RSSI reaches its maximum value, the pedestrian arrives at the reference point. Therefore, the sum of the step length, *L*_sum_, between the two reference points can be known.

As shown in Figure 2, the sum step length *L*_sum_ between the start point and the end point in this example is *L*_2_ + *L*_3_ + *L*_4_. In the traditional PDR, PCP is the empirical value. In DRBM, PCP is updated through the real distance *D* and *L*_sum_ and no longer relies on the empirical value. DRBM named this update method as linear update.

(2) $$\begin{array}{c} s_{t+1}=s_{t}\times \frac{D}{L_{sum}}. \end{array}$$

## 4. SHAKF-PU: SHAKF-Based PCP Update Mechanism

In Equation (1), the setting of PCPs affects the accuracy of the SLE. Equation (2) gives the linear update formula, *s*_*t* + 1_ can be regarded as the true value *Rs* of this positioning, and *s*_*t*_ can be regarded as the estimated value of this positioning.

In the actual operation, the *s* value for each update is different. It means that the estimated value is different from the true value, which causes distance errors. When the estimated value is not equal to the true value, the distance error occurs.

When the estimated value can be adjusted to make the estimated value close to the true value, the distance error can be reduced compared with the linear update. SHAKF-MU uses SHAKF to adjust the estimated value. Because SHAKF has the characteristics of forecasting based on historical data, the estimation of *s* value is close to the true value, *Rs*, in order to reduce the distance error.

(3) $$\begin{array}{c} Rs=s_{t}\times \frac{D}{L_{\text{sum}}}, \end{array}$$

(4) $$\begin{array}{c} s_{t+1}=\text{SHAKF}\left(Rs,s_{t}\right). \end{array}$$

To estimate the PCP value by SHAKF, the true value *Rs* is the measured value, and *s*_*t*_ is the current predicted PCP value. They are the inputs for SHAKF to estimate the next predicted PCP value *s*_*t*+1_.

Equation (5) is the base Kalman filter system equation [3]:

(5) $$\begin{array}{c} X_{t}=FX_{t-1}+HU_{t}+BW_{t}. \end{array}$$

In Equation (5), *t* is the time variable, *X* is the predicted value, *U* is the system control variable, *B*, *F*, and *H* are the system parameters, and *W* is the noise.

The process formula of SHAKF [11, 13] shows as follows:

(6) $$\begin{array}{c} X_{t\left|t-1\right.}=FX_{t-1\left|t-1\right.}+HU_{t}+Bq_{t-1}, \end{array}$$

(7) $$\begin{array}{c} P_{t\left|t-1\right.}=FP_{t-1\left|t-1\right.}F^{T}+BQ_{t-1}B^{T}, \end{array}$$

(8) $$\begin{array}{c} Kg_{t}=P_{t\left|t-1\right.}H^{T}/\left(HP_{t\left|t-1\right.}H^{T}+R_{t-1}\right), \end{array}$$

(9) $$\begin{array}{c} e_{t}=Z_{t}-HX_{t\left|t-1\right.}-r_{t-1}, \end{array}$$

(10) $$\begin{array}{c} X_{t\left|t\right.}=X_{t\left|t-1\right.}+Kg_{t}e_{t}, \end{array}$$

(11) $$\begin{array}{c} P_{t\left|t\right.}=\left(I-kg_{t}H\right)P_{t\left|t-1\right.}. \end{array}$$

In these equations, *F*, *H*, and *B* are system parameters, and *I* is the identity matrix. *X*_*t*|*t*−1_ is the result of using the previous state prediction, *X*_*t*|*t*−1_ is the result of the system in the previous state, and *P*_*t*|*t*−1_ is the covariance corresponding to *X*_*t*|*t*−1_. *P*_*t*−1|*t*−1_ is the covariance corresponding to *X*_*t*−1|*t*−1_, *Kg* is Kalman gain, and *e*_*t*_ is the residual. *Q* is the covariance of the predicted value, and *R* is the covariance of the measured value. The real value *Rs* is input as the measured value *Z*, and SHAKF gives the output predicted value *X* as the new estimated value *s*_*t*+1_.

*Q* is regarded as a weight between the measured value and the predicted value. The large *Q* value shows the measured values are trustable. The small *Q* value shows the high confidence of the predicted values. *R* is used to control the speed of convergence. The small R values lead to the fast system converges.

In CKF, *Q* and *R* remain constant after setting the initial value. If *Q* and *R* are not set properly, the effect may be worse than the effect without filtering. In SHAKF, *Q* and *R* can be updated in real time through a recursive estimator of time-varying noise statistics. It solves the problem that *Q* and *R* may be manually set incorrectly. Because *Q* and *R* can be updated automatically, it is more flexible than CKF.

The recursive estimator of time-varying noise statistics shows as follows [11, 13]:

(12) $$\begin{array}{c} d_{t}=\frac{1-b}{1-b^{t+1}},0<b<1, \end{array}$$

(13) $$\begin{array}{c} qt=\left(1-d_{t-1}\right)q_{t-1}+d_{t-1}\left(X_{t\left|t\right.}-FX_{t-1\left|t-1\right.}\right), \end{array}$$

(14) $$\begin{array}{c} Q_{t}=\left(1-d_{t-1}\right)Q_{t-1}+d_{t-1}\left(Kg_{t}e_{t}{e_{t}}^{T}Kg^{T}+P_{t\left|t\right.}-FP_{t-1\left|t-1\right.}F^{T}\right), \end{array}$$

(15) $$\begin{array}{c} r_{t}=\left(1-d_{t-1}\right)r_{t-1}+d_{t-1}\left(Z_{t}-HX_{t\left|t-1\right.}\right), \end{array}$$

(16) $$\begin{array}{c} R_{t}=\left(1-d_{t-1}\right)R_{t-1}+d_{t-1}\left(e_{t}{e_{t}}^{T}-HP_{t\left|t-1\right.}H^{T}\right). \end{array}$$

In these equations, *b* is the attenuation parameter. *d* is the weighting coefficient, and *q* and *r* are the noise factors. The measured value *Z* of SHAKF is the input, and the predicted value *X* is the output. *F*, *H*, *B*, *I*, and *b* are system parameters that need to be set.

## 5. Enhanced SLE Based on SHAKF-PU

SHAKF-PU is designed to compute the accurate estimated value *s* to be close to the true value *Rs*.  Algorithm 1 shows the new SLE is enhanced based on SHAKF-PU.

First, the real distance *D* between the start point and the endpoint is known. Through the RSSI of the start point and the endpoint, it can be known that the reference point position state, *RPstate*, is before the start point, between the start point and the endpoint, or after the endpoint.

When the position is before the starting point (*RPstate* = −1), the sum step length *Lsum* is always 0. When the position is between the starting point and the ending point (*RPstate* = 0), the calculated step length *Lsum* is added to the sum of the current step length. When the position is after the endpoint (*RPstate* = 1), PCP is updated.

When PCP is updated, the true value *Rs* is obtained. Then *Rs* is the input as the measured value *Z* into SHAKF-PU to obtain the predicted value *X*. The predicted value *X* is the output as the new estimated value *s*. Because SHAKF has the characteristic of predicting the direction of historical data, as long as the number of positioning is sufficient, the estimated value s gets close to the true value *Rs*, and the distance error becomes small.  Algorithm 2 shows the process of SHAKF-PU as follows:

In Algorithm 2, *F*, *H*, *B*, *I*, and *b* need to be given parameter values; the input is *Z*, and the output is *X*. In SHAKF-PU, it sets *F* = 1, *H* = 1, *B* = 1, *I* = 1, *b* = 0.99. *Rs* is the input as the measured value *Z*, and *s* is the output as the predicted value *X*.

## 6. Experimental Results

### 6.1. Experiment Setting

The experimental equipment in this paper includes nine-axis sensors and Bluetooth chips. The nine-axis sensor is MPU9250. The Bluetooth chip is a low-power Bluetooth chip produced by Broadcom, and the model is BCM92073X_LE_KIT. The experimental environment is in the corridor of the National Taipei University building. The distance between the two Bluetooth chips at the receiving end is 12 m. Hold a nine-axis sensor and two Bluetooth chips as the transmitter. The nine-axis sensor collects data and converts it into vertical acceleration on the ground through quaternion. The Bluetooth chip collects RSSI, and the transmitting frequency between Bluetooth chips is 10 times per second. One end of the Bluetooth chip is used as the starting point, and the other end is used as the endpoint.

This experiment compares four ways of updating PCP: (1) Linear: linear updating; (2) AVG (5): the average of the last five PCP samples; (3) CKF: classical KF; (4) AKF: SHAKF. When the estimated value of PCP is close to the true value, the distance error is reduced. CKF presents those relative works that adopt the Kalman filter for PCP updates [3–5].

### 6.2. Distance Error Comparisons

The difference between the estimated value of PCP and the true value causes distance error. The distance error is the difference between the real distance *D* and the sum of the step length *L*_*sum*_.

(17) $$\begin{array}{c} \text{Distance error}=\left|D-L_{\text{sum}}\right|. \end{array}$$

In the experiment, the true distance *D* is defined as 12 m. When the difference between the estimated value of PCP and the true value is large, the distance error is also large. This section compares the distance errors of linear update, AKF, average filtering, and CKF.

Figure 3 shows that linear update and average filtering are worse than CKF and AKF in general. After the number of positioning times is above 5, AKF is better than KF. So, AKF is the best of the four methods in general.

To compare AKF and CKF, Figure 4 shows that the cumulative error of AKF is smaller than CKF when the number of positioning times reaches more than 10 times. The performance of average filtering in this experiment is very close to AKF.  Figure 5 focuses on comparing AKF and AVG (5) to compare them effectively.

Figure 5 shows that the cumulative distance error of AKF is smaller than AVG (5) at the 17th, 18th, and 20th positioning, but AKF is higher than AVG (5) filtering at the 19th positioning. To compare them with more experiment results, we repeated this experiment five times to confirm that AKF is indeed better than average filtering, as shown in Figure 6.

From Figure 6, it is clear that after the cumulative distance error of five experiments is added and averaged, the cumulative distance error of AKF is less than that of the average filter. It shows that AKF is indeed effective in predicting PCP. When the number of positioning is higher than 10 times, the cumulative distance error of AKF is the smallest compared with the other three.

Table 1 shows that the distance error of AKF is less than average filtering, CKF, and linear update. The average distance error of AKF is 2.36 m. It is 0.11 m less than the average filter, 0.42 m less than the CKF, and 0.65 m less than the linear update. In summary, AKF is indeed the best of the four update methods. The numbers in bold are best results in the four methods, and AKF is the best in the results.

### 6.3. Distance Error in Different Positioning Times

AKF has the characteristics of historical data trend prediction. As the number of positioning times increases, the distance error should be smaller. Four hundred positionings were performed in this section. This experiment shows the distance error of PCP is reduced by AKF when the number positioning times increases.

Figure 7 shows that AKF is unstable when the number of positioning times does not exceed 10 times. After the number of positioning times exceeds 10 times, the distance error of AKF is the smallest of the four methods. Besides, as the number of positioning increases, the distance error of AKF becomes small because of its accurate prediction.

Table 2 shows that when AKF has only 20 positioning times, the average distance error is 2.33 m. When the number of positioning times becomes 400, the average distance error is 2.16 m. This shows that AKF's prediction is getting accurate, and the distance error is getting smaller. The numbers in bold are best results in the four methods, and AKF is the best in most of the results.

In addition, the standard deviation of AKF positioning error decreases as the times of positioning increase. The reduction of the standard deviation means that the fluctuation of the positioning error is reduced because the estimated value given by AKF is getting close to the true value.

When the number of positioning times is less than 40, the standard deviation of the average filtering is smaller than AKF. Because the characteristic of average filtering is smoothing, it is inevitable that the standard deviation can be reduced. When the number of positioning times becomes more than 100, since the predicted trend of AKF starts to approach the true value, the advantage of the average filter no longer exists.

Compared with the original linear update method, AKF has reduced the distance error by 24.86%. In the meanwhile, average filtering reduces the distance error by 19.98%, and CKF reduces the distance error by 13.10%. Therefore, by adopting SHAKF, SHAKF-PU provides the best positioning accuracy than the linear update, the average, and the Kalman filter.

### 6.4. Experimental Result Summary

According to the experimental results, PCP filtering methods are better than the linear update. AKF is slightly inferior to CKF when the number of positioning times is less than 10, and the effect is close to the average filtering. Between 10 and 20 positioning times, AKF and average filtering are close, while KF performs poorly. When the number of positioning becomes more than 20, AKF performance is the best of the three.

AKF has the characteristic of forecasting based on historical data. When the number of positioning time increases, the distance error becomes small. When the number of positioning time is 20, the average distance error is 2.33 m. When the number of positioning time becomes 400, the average distance error is reduced to 2.16 m. In addition, the standard deviation of distance error also decreases when the number of positioning times increases. This shows the AKF prediction is getting close to the true value, and the fluctuation of the distance error is getting small.

Compared to the linear update proposed by DRBM, AKF reduces the distance error by 24.86%, and the effect is obvious. The experiment also compares the average filter and CKF, which reduces the distance error by 19.98% and 13.10%, respectively. Thus, SHAKF-MU is the best choice in PCP update mode.

## 7. Conclusion

This paper proposes SHAKF-MU that adopts SHAKF to update PCP. Based on the characteristic of SHAKF to predict the trend of historical data, the estimated PCP value is getting close to the true value, and the distance error can be reduced. The experimental results show that SHAKF-MU has the smallest distance errors. Compared with the original linear update, SHAKF-MU reduced the distance error by 24.86%. The average and Kalman filter only reduced the distance errors by 19.98% and 13.10%, respectively. In addition, because SHAKF has predictive characteristics, the distance error becomes small as the number of positioning times increases. When the number of positioning times is 20, the average distance error for every 12 m walked is 2.33 m. When the number of positioning times is 400, the average distance error for every 12 m walked is 2.16 m. Thus, SHAKF-PU provides better results with 400 positioning times than 20 times without cumulative errors.

## Figures and Tables

**Figure 1:** Step state value.

**Figure 2:** Sum of the step lengths.

**Figure 3:** The process of distance error in four update methods.

**Figure 4:** Cumulative distance error of four update methods.

**Figure 5:** Cumulative distance error of AKF and AVG (5).

**Figure 6:** Cumulative distance error over five experiments.

**Figure 7:** Average distance error.

**Algorithm 1:** Enhanced SLE based on SHAKF-PU.

**Algorithm 2:** SHAKF-PU.

**Table 1:** Cumulative distance errors in five 20-times tests.

	AKF	AVG (5)	CKF	Linear
1st	**49.52312**	49.97666	56.33625	69.66213
2st	**44.38289**	48.17956	60.03855	55.87052
3st	**49.17905**	50.18651	59.16382	54.69721
4st	**46.21081**	49.91435	50.06121	60.90114
5st	**46.82417**	48.89955	52.34962	60.08161
Average	**47.22401**	49.43133	55.58989	60.24252

**Table 2:** Sum, average, and standard deviation (SD) of distance errors in 20–400 times.

Experiments		AKF	AVG (5)	CKF	Linear
20	Sum	**46.6**	55.5	57.3	62.5
	Average	**2.33**	2.78	2.86	3.13
	SD	1.9	**1.77**	2.23	2.41

40	Sum	**89.3**	96.2	96.5	124
	Average	**2.23**	2.41	2.41	3.09
	SD	1.64	**1.59**	1.9	2.33

100	Sum	**220**	239	280	285
	Average	**2.20**	2.39	2.8	2.85
	SD	**1.50**	1.73	1.97	2.49

200	Sum	**436**	456	502	555
	Average	**2.18**	2.28	2.51	2.78
	SD	**1.17**	1.62	1.92	2.47

400	Sum	**863**	919	998	1,148
	Average	**2.16**	2.3	2.5	2.88
	SD	**1.15**	1.6	1.95	2.38

## Data Availability

The data presented in this study are available on request from the first author.
